# Preoperative ICG Test to Predict Posthepatectomy Liver Failure and Postoperative Outcomes in Hilar Cholangiocarcinoma

**DOI:** 10.1155/2021/8298737

**Published:** 2021-02-23

**Authors:** Min Li, Jie Wang, Jieqiong Song, Feng Shen, Lujun Song, Xiaoling Ni, Tao Suo, Han Liu, Ming Zhong, Houbao Liu

**Affiliations:** ^1^Department of General Surgery, Zhongshan Hospital, Fudan University, 180, Fenglin Road, Shanghai 200032, China; ^2^Department of Critical Care Medicine, Zhongshan Hospital, Fudan University, 180, Fenglin Road, Shanghai 200032, China; ^3^Department of Medical Oncology, Zhongshan Hospital, Fudan University, 180, Fenglin Road, Shanghai 200032, China

## Abstract

Preoperative evaluation of hepatic functional reserve in patients with hilar cholangiocarcinoma (hCCA) has vital clinical significance for prevention of posthepatectomy liver failure (PHLF) and mortality. The aim of the present study was to evaluate the clinical significance of the indocyanine green retention rate at 15 minutes (ICG R15) and related factors of postoperative outcomes in patients with hCCA. 147 patients who scheduled for hCCA resection underwent a preoperative ICG test between May 2015 and May 2020 and were prospectively analyzed. Single-factor analysis was used to evaluate the risk factors for PHLF and postoperative outcomes in hCCA. After univariate analysis, significant differences in ICG R15 were found between the PHLF group and the liver function recovered well (LFRW) group (*P* ≤ 0.05). In terms of postoperative complications, ICG R15 was also a risk factor for moderate-to-severe postoperative complications. Preoperative ICG R15 was significantly associated with PHLF and moderate-to-severe postoperative complications. ICG R15 may become an ideal clinical indicator for the evaluation of liver function reserve before hCCA and can better predict the postoperative complications.

## 1. Introduction

Cholangiocarcinomas (CC) are the third most common tumor resulting in death [1, 2]. In general, CC can be divided into three subtypes: intrahepatic or peripheral CC (ICC), hilar cholangiocarcinoma (hCCA), or Klatskin tumor and distal ICC [3]. hCCA comprises over 60% of all CC, which is a rare and highly malignant cancer with a poor prognosis [2]. Multiple treatment strategies are available for hCCA, including hepatic resection, liver transplantation, radiofrequency ablation, and radioembolization [4]. Surgery should always be considered the best treatment option and maybe the only available curative therapy for patients with early-stage hCCA [5]. However, hepatic resection still remains the major surgical treatment for hCCA, especially in Asia, where a shortage of liver grafts greatly restraining its clinical application [1, 5].

With recent advances in surgical technology and perioperative management, postoperative liver failure still occasionally occurs in cases of hepatic resection [6]. So, it is critical to evaluate liver function for hepatic resection. The conventional approaches used to assess liver function include both quantitative and passive liver function assessment. Quantitative liver function assessment mainly includes the indocyanine green (ICG) clearance test, and passive liver function assessment includes scoring systems, such as the Child-Pugh classification and model for end-stage liver disease (MELD) score, and multiple clinical parameters, such as aminotransferase levels, serum albumin, the international normalized ratio (INR), and serum bilirubin levels [7, 8]. The Child-Pugh classification has been widely used to evaluate the quality of the liver for years [9]. In recent years, two significant studies drew conclusions: class A patients experienced a higher operative mortality rate than class B and class C patients [10]. However, Child-Pugh A patients could sometimes have different levels of hepatic functional reserve. Therefore, a more accurate preoperative assessment of the patient's liver function is vital to avoid postoperative hepatic failure and mortality [11, 12].

Without the limitations of the above passive liver function assessment, quantitative tests of liver function have an advantage in severity assessment, long-term prognosis, and surgical risk evaluation of liver disease [13]. The ICG clearance test has been identified as the most widely used quantitative assessment of preoperative liver function test [14]. Moreover, it is a noninvasive test that can be performed at the patient's bedside [15]. ICG is a water-soluble fluorescent cyanine dye, and its blood clearance has been identified as an indirect evaluation of hepatic functional reserve before hepatectomy [16]. The ICG retention rate at 15 minutes (ICG R15) has been proven to be positively correlated with posthepatectomy liver failure and morbidity after hepatic resection in patients with liver disease [8]. Previous studies have also shown that clearance is impaired and hepatectomy may increase the risk of postoperative hepatic injury when ICG R15 is above 14% after major hepatectomy [17].

Postoperative hepatic dysfunction remains a primary cause of early postoperative mortality in patients undergoing hCCA resection. Therefore, adequate preoperative evaluation of the patient's hepatic functional reserve has vital clinical significance. However, current data on the value of preoperative ICG clearance testing to predict the development of PHLF in hCCA are scarce, and most of the studies have been limited to hepatic carcinoma. Besides, there are few reports on related factors of postoperative outcomes in patients with hilar cholangiocarcinoma. The aim of the present study was to evaluate the clinical significance of ICG R15 and related factors of postoperative outcomes in patients with hCCA in our hospital.

## 2. Materials and Methods

### 2.1. Patients

The study protocol was approved by the institutional ethical committees of Zhongshan Hospital. Between May 2015 and May 2020, a consecutive series of 147 cases who underwent R0 resection for hCCA in the Department of Surgery were included in this prospective study. All patients gave written informed consent. The final diagnosis of hCCA was confirmed by the postoperative pathology of the operative specimens. The inclusion criteria were (1) preoperative clinical diagnosis of Bismuth II, III, or IV, (2) no definitely extrahepatic metastasis from comprehensive preopreative examination, and (3) no neoadjuvant chemotherapy before hepatectomy. The exclusion criteria were (1) preoperative clinical diagnosis of Bismuth I, (2) patients or their families refusing the surgery, (3) associated comorbidities such as cirrhosis or severe abnormal liver function before surgery, and (4) other serious comorbidities that could not tolerate surgery.

### 2.2. Definitions

As different definitions of posthepatectomy liver failure (PHLF) have been used, the standard of PHLF in our study accorded with the criteria proposed by the International Hepatic Surgery Research Group (ISGLS) in 2011, which is simple and easily applicable in clinical practice [18]. Increased INR and concomitant hyperbilirubinemia on or after postoperative day 5 were diagnosed with PHLF. According to the normal limits of our laboratory, bilirubin > 17.1 *μ*mol/L was taken as hyperbilirubinemia, and INR was increased when it was over 1.20. However, some distinct causes for the clinical and biochemical changes, such as biliary obstruction, should be ruled out. For patients with preoperatively increased INR or hyperbilirubinemia, PHLF should be defined by hyperbilirubinemia and increased INR on or after postoperative day 5 compared with the preoperative indicators. In addition, hyperbilirubinemia in combination with impaired coagulation function such that fresh frozen plasma should be employed on or after postoperative day 5 to maintain normal INR is also considered to be PHLF. The severity of PHLF is mainly divided into the following three grades: grade A, with abnormal laboratory indicators and requiring no special intervention in clinical management; grade B, with abnormal laboratory indicators and requiring clinical intervention rather than invasive procedures (e.g., infusion of fresh frozen plasma, albumin, diuresis, and noninvasive ventilation); and grade C, with abnormal laboratory indicators and requiring invasive procedures, including hemodialysis, intubation, mechanical ventilation, artificial liver, and liver transplantation [18].

### 2.3. Preoperative Biliary Drainage

After admission, the laboratory examination should be completed, and preoperative percutaneous transhepatic biliary drainage (PTBD) would be applied for patients with high bilirubin levels, cholangitis, prolonged prothrombin time, and intrahepatic bile duct dilatation (diameter > 3 mm) by B-ultrasound. The patient was placed in the supine position, and appropriate segmental duct was punctured under ultrasound guidance. After successful intrahepatic bile duct puncture, 1 : 1 contrast agent was injected to show intrahepatic bile duct; the guidewire was used to penetrate the intrahepatic bile duct. Then, the puncture site was cut to expand the puncture channel, and a three-piece set of PTBD was exchanged and injected through the outer cannula. 1 : 1 contrast agent was injected again, external drainage tube was placed through the outer cannula by means of a guidewire exchange. After the angiography confirmed that the drainage tube was in place, the drainage tube was fixed and connected to the drainage bag.

### 2.4. ICG Test

All patients fasted for 6 hours and then received the ICG test the day before surgery. After the patient's height, weight, and other values were inputted into the analyzer, a single bolus dose of 0.5 mg/kg ICG (dissolved in 10 mL sterile water; Dandong Yichuang Pharmaceutical Co., Ltd., Liaoning, China) was administered intravenously into a peripheral vein of patients who were in a supine position within 10 seconds. Venous blood samples were drawn and read with a pulse spectrophotometer at 805 nm at 15-minute intervals. The results were displayed as ICG R15 after injection. It should be noted that in patients with jaundice, the ICGR15 should be detected when serum bilirubin level was back to normal after preoperative biliary drainage.

### 2.5. Surgical Procedures

All the procedures were performed by an experienced surgeon. All patients in our study underwent tumor removal via a curved incision under the right costal margin. Preoperative abdominal computed tomography (CT), multislice spiral computed tomographic angiography, and magnetic resonance cholangiopancreatography were routinely performed for patients to assess tumor location, biliary tree, vascular variation, or the presence of extrahepatic disease. An initial surgical exploration was performed, and patients without distant metastasis would undergo further assessment of resectability. If resectability was confirmed, the entire tumor, including the gallbladder, cystic duct, and extrahepatic bile duct, was removed, and lymph node dissection of the celiac axis, common hepatic artery, and hepatoduodenal ligament was performed to obtain a surgical margin-negative (R0) resection. We suggested that the bile duct should be resected at least 10 mm above the tumor if possible, and frozen section analysis of resection margins was applied to guide resection in the meantime. Extended resection was implemented when the resection margins were initially positive. The extent of liver resection was determined according to the size, location, and proximity to peripheral vascular structures of the tumor [8]. The choice of whether to perform extensive hepatic resection depended on the function and the volume of the remnant liver. The anaesthetist attempted to maintain central venous pressure at low levels during the entire surgery. The intermittent Pringle maneuver or selective inflow occlusion was performed selectively during extensive hepatectomy if necessary. Roux-en-Y hepaticojejunostomy was performed for the biliary after resection reconstruction. The resected liver volume was calculated by the water volume displacement method.

### 2.6. Statistics

Classified variables were expressed as absolute numbers and percentages, while continuous variables were expressed as medians and ranges. Data analysis was performed using SPSS 20.0 (IBM, USA). The classified variables between groups were analyzed using the Chi-square test or Fisher's exact test, as appropriate. Continuous variables between groups were analyzed using the unpaired *t*-test, if the data is normally distributed. *P* ≤ 0.05 was considered statistically significant.

## 3. Results and Discussion

### 3.1. All Patients' Characteristics

A total of 147 patients (81 male and 66 female) who met the inclusion criteria were included in this study with a median age of 64 (34-80) years and median weight of 59 (37-95) kg, and 19 patients (12.93%) had a history of chronic hepatitis. The patients' characteristics, preoperative laboratory results, and related data are shown in Table 1. Most patients (*n* = 84, 57.14%) were Childs A, while 63 patients were Childs B (42.86%). The preoperative median platelet count, serum albumin, serum bilirubin, alkaline phosphatase, G-glutamyl transferase, INR, and serum creatinine were 214 (63 − 412) × 109/L, 40 (32-47) g/L, 9.4 (4.5-16.9) mg/dL, 230 (41-1389) U/L, 330 (19-1977) U/L, 0.96 (0.83-1.25), and 60 (38-103) mg/dL, respectively. The preoperative median plasma disappearance rate (PDR) and ICG R15 values were 13.9 (3.2-46.6) %/min and 12.2 (0.5-61.9) %, respectively. The 30-day and 90-day postoperative mortality rates were 3 (2.04%) and 2 (1.36%), respectively.

### 3.2. Clinical and Pathology Data of the Patients

The relevant intraoperative data are summarized in Table 2. The median operation time was 465 (79-950) minutes with a median intraoperative blood loss of 350 (40-1200) mL. The median blood transfusion included 0 (0-6) units of concentrated red blood cells and 0 (0-800) mL plasma. The median obstructive time of the portal vein was 0 (0-52) min. The median length of hospital stay was 23 (7.0-49.5) days. The median volume of resected liver was 216 (55.0-1611.0) cm^3^. Microscopically, more than 95% of tumors (140/147) were conventional-type adenocarcinomas, mostly well to moderately differentiated. Seven patients (4.76%) were diagnosed with papillary carcinoma.

### 3.3. Clavien's Classification of Complications

According to Clavien's classification of complications, postoperative complications account for 92.52% of patients undergoing R0 resection, and Clavien grade IV was not observed in our study, while major complications (including Clavien grades IIIb and V) were encountered in 4 patients (2.72%). Clavien's classification of complications is shown in Table 3. In most cases, most of the postoperative complications were mild or moderate, and Clavien grade I accounted for 39.46% of all the complications. Clavien grade I complications included 20 (13.61%) patients with pain, 18 (12.24%) patients with vomiting, 11 (7.48%) patients with pleural effusion, 6 (4.08%) patients with ascites, and 3 (2.04%) patients with fever, who recovered without need for interventional treatment. In addition, Clavien grade II accounted for 40.82% of all complications, including 37 (25.17%) patients with pleural effusion, 7 (4.76%) patients with ascites, 6 (4.08%) patients with fever, 4 (2.72%) patients with pulmonary embolism, 3 (2.04%) patients with biloma, and 3 (2.04%) patients with liver abscess, who required pharmacological treatments such as antibiotics and total parenteral nutrition. Moreover, there were 14 (9.52%) Clavien grade IIIa and 1 (0.68%) Clavien grade IIIb complications in our research, respectively. The Clavien grade IIIa complications included 8 (5.44%) cases with pleural effusion and 6 (4.08%) cases with ascites who received ultrasound-guided drainage separately; the Clavien grade IIIb complication included 1 case with incisional hernia who received hernia repair treatment. Furthermore, 3 patients with Clavien grade V complications were diagnosed with intra-abdominal hemorrhage after surgery and received a series of treatments, including digestive angiography, intravascular embolization, tracheotomy, or hemodialysis.

### 3.4. Preoperative ICG Clearance Is Associated with PHLF

The postoperative liver function was evaluated according to the criteria proposed by ISGLS. The associated characteristics, preoperative laboratory results, and some clinical data of the patients in the PHLF group and the liver function recovered well (LFRW) group are shown in Table 4. The liver function of 93 patients (63.27%) recovered well after surgery, and 54 patients (36.73%) were considered to be PHLF. Patients with PHLF included 21 cases of grade A (38.89%), 27 cases of grade B (50%), and 6 cases of grade C (11.11%).

### 3.5. Correlation of Postoperative Outcomes and Clinical Characteristics

To further assess the factors affecting postoperative complications, we divided postoperative complications into two groups: a minor complication group (including Clavien grade I) and a moderate-to-severe complication group (including Clavien grades II, IIIa, IIIb, IV, and V). The patients' associated characteristics, preoperative laboratory results, clinical data, and postoperative liver function in the minor group and the moderate-to-severe group are shown in Table 5.

## 4. Discussion

hCCA is a highly malignant cancer, and surgery may be the only available curative therapy for patients. Currently, the gold standard for hCCA is major liver resection combined with extrahepatic bile duct resection in most centers, which can increase the R0 resection rate and improve the long-term survival rate [2]. However, PHLF after major hepatectomy is difficult to treat and has a high mortality rate. Considering the risk of PHLF, it is important to perform an accurate assessment of preoperative liver function reserve. However, current data on the value of preoperative ICG clearance testing to predict the development of PHLF are scarce, and studies have been limited to hepatic carcinoma.

In general, the assessment of liver functional reserve is mainly divided into passive liver tests and dynamic quantitative liver function tests. Passive liver function tests mainly include biochemical parameters and clinical grading systems. Commonly available laboratory tests include alanine transferase (ALT) and aspartate transferase (AST), which closely related to the extent of hepatocellular predominant disorders [19]. The plasma concentrations of albumin and coagulation factors are routinely used as indirect indicators of liver function [20]. Coagulation time gives a reliable evaluation of acute alterations in the synthetic function of the liver [13]. In addition, the frequently used clinical grading systems include the Child-Pugh and MELD scoring systems. The Child-Pugh score is always used to assess the prognosis of chronic liver disease and the necessity of liver transplant [8]. The MELD scoring system also has inherent limitations, including vulnerability to variations and the absence of clear-cut discriminant values [21–23]. As a result, neither the Child-Pugh nor the MELD score can be used to evaluate the risk of hepatic failure for patients with noncirrhotic livers or estimate small changes in the liver metabolic capacity [13, 24]. In addition, biochemical parameters and clinical grading systems can provide only indirect information about liver function.

Therefore, especially for some patients without cirrhosis, objective liver function assessment is needed in addition to clinical judgment. Without the limitations of the above liver function tests, quantitative tests of liver function have an advantage in severity assessment, long-term prognosis, and surgical risk evaluation of liver disease [13]. The commonly used quantitative tests of liver function include the ICG clearance test, galactose elimination capacity, and monoethylglycinexylidide test [13]. In clinical practice, the ICG clearance test has become the most widely used dynamic quantitative test of liver function due to its advantages of safety, effectiveness, noninvasiveness, and easy operation. Some studies have also revealed that the ICG test could offer early and sensitive evaluation of liver dysfunction in patients with acute liver failure [25]. Therefore, the ICG test is considered to be one of the ideal methods for accurate perioperative assessment of liver function, and it has become the most widely used quantitative test of dynamic liver function.

To date, there are few reports on the ICG R15 test in predicting the prognosis of acute liver failure in hCCA. This research mainly evaluated the clinical significance of ICG R15 in predicting PHLF in patients with hCCA in our hospital. In our research, we found that postoperative complications account for 92.52% of patients undergoing R0 resection; most of the postoperative complications were mild or moderate while major complications were encountered in 2.72% of patients. The incidence of postoperative complications was reported to be 81.0% in Masato's research, which was similar to our research [26]. 36.73% patients undergoing hCCA resection were considered to be PHLF, which was slightly higher than that previously reported [26]. The associated characteristics, preoperative laboratory results, and some clinical data of the patients were compared between the PHLF group and the LFRW group. We found there was no significant difference in age, sex, history of chronic hepatitis, serum bilirubin, serum albumin, INR, operation time, intraoperative blood loss, volume of resected liver, or surgical method between the PHLF group and the LFRW group (*P* > 0.05). However, preoperative ICG R15 was significantly associated with PHLF in hCCA (*P* ≤ 0.05). At the same time, another clinical research showed ICG clearance test was a valuable tool to identify patients at risk of developing PHLF after liver resection [27]. To further assess the factors affecting postoperative complications, we found there was a significant difference in ICG R15 between the minor group and the moderate-to-severe group (*P* ≤ 0.05). There was no significant difference in age, sex, history of chronic hepatitis, serum bilirubin, serum albumin, INR, operation time, intraoperative blood loss, volume of resected liver, or surgical method between the minor group and the moderate-to-severe group (*P* > 0.05). Therefore, the above results demonstrated that ICG R15 was a risk factor for moderate-to-severe postoperative complications. Some previous studies also found that ICG clearance test enables prediction of postoperative complications after hepatic resection [28].

Expect for the research findings, there are also some research limitations in the present study. First, this was a retrospective observational study with inevitable biases for patient selection, and some vital clinical data could not be obtained. Selection bias was minimized in this study by analyzing a consecutive series of patients who were treated by a single surgeon in a single institute. Some vital clinical data remains to be further studied in future research. Second, this study did not provide long-term follow-up data of patients, so further long-term studies are needed. Third, the study lacked sufficient data for the low incidence rate of hCCA, so larger trials are needed to better evaluate the clinical efficacy and safety of ICG R15.

ICG R15 may become an ideal clinical indicator for the evaluation of liver function reserve before hCCA and better predict the recovery of postoperative liver function. If there is an abnormality in the liver function reserve before surgery, the extent of liver excision should be carefully determined during the operation, and the postoperative liver function and complications should be closely observed after surgery. If necessary, intervention should be performed as soon as possible to prevent postoperative PHLF and serious complications such as liver function failure.

## 5. Conclusions

hCCA is a rare and highly malignant cancer that continues to present formidable challenges in preoperative diagnosis, evaluation, and postoperative management. We found that preoperative ICG R15 was significantly associated with PHLF and moderate-to-severe postoperative complications. As a consequence, in patients who are potentially resectable, careful preoperative assessment, potentially including the ICG clearance test, biliary drainage, and comprehensive preoperative geriatric assessment, should be carried out to prevent postoperative PHLF or serious complications. However, due to the relatively lower incidence and surgical R0 resection rate of hCCA, the number of cases included in this study was small. The postoperative follow-up time was not long enough to find long-term complications. Therefore, further studies with more patients and longer follow-up times would be more valuable and meaningful.

## Figures and Tables

**Table 1:** Demographics and preoperative data of the 147 patients included in the study.

Demographics and preoperative data	
Sex, *N* (%)	
Male	81 (55.10)
Female	66 (44.90)
Age, years (range)	64 (34-80)
Weight (kg)	59 (37-95)
History of chronic hepatitis, *N* (%)	
Hepatitis B	16 (10.88)
Hepatitis C	3 (2.04)
Child-Pugh score, *N* (%)	
A	84 (57.14)
B	63 (42.86)
Platelet count (10^9^/L)	214 (63-412)
Serum albumin (g/L)	40 (32-47)
Serum bilirubin (mg/dL)	9.4 (4.5-16.9)
Alkaline phosphatase (U/L)	230 (41-1389)
G-glutamyl transferase (U/L)	330 (19-1977)
INR	0.96 (0.83-1.25)
Serum creatinine (mg/dL)	60 (38-103)
PDR (%/min)	13.9 (3.2-46.6)
ICG R15 (%)	12.2 (0.5-61.9)
30 day postoperative mortality	3 (2.04%)
90 day postoperative mortality	2 (1.36%)

Values are presented as *n* (%) or median (range). *INR*: international normalized ratio; *PDR*: plasma disappearance rate; *ICG R15*: indocyanine green retention rate at 15 minutes.

**Table 2:** Clinical and pathology data of 147 patients who received R0 resection.

Data assessed	
Operation time (min)	465 (79-950)
Intraoperative blood loss (mL)	350 (40-1200)
*Blood transfusion*	
Concentrated red blood cells (units)	0 (0-6)
Plasma (mL)	0 (0-800)
Obstructive time of portal vein (min)	0 (0-52)
Length of hospital stay (days)	23 (7.0-49.5)
Volume of resected liver (cm^3^)	216 (55.0-1611.0)
*Histopathology (%)*	
Adenocarcinoma	140 (95.24)
Papillary carcinoma	7 (4.76)

Values are presented as *n* (%) or median (range).

**Table 3:** Clavien's classification of complications.

Clavien's grade	Complication	*N* (%)
I	Pain	20 (13.61)
	Vomiting	18 (12.24)
	Pleural effusion	11 (7.48)
	Ascites	6 (4.08)
	Fever	3 (2.04)
II	Pleural effusion	37 (25.17)
	Ascites	7 (4.76)
	Fever	6 (4.08)
	Pulmonary embolism	4 (2.72)
	Biloma	3 (2.04)
	Liver abscess	3 (2.04)
IIIa	Pleural effusion	8 (5.44)
	Ascites	6 (4.08)
IIIb	Incisional hernia	1 (0.68)
IV	No	0 (0.00)
V	Intra-abdominal hemorrhage	3 (2.04)
All		136 (92.52)

**Table 4:** Postoperative data between PHLF group and LFRW group.

Factor	Group	Result	*P* value
Age, years	LFRW	64 (34-78)	0.958
	PHLF	63 (50-80)	
Sex, *N*			
Male	LFRW	51	0.933
	PHLF	30	
Female	LFRW	42	
	PHLF	24	
Hepatitis, *N*			
Yes	LFRW	11	0.603
	PHLF	8	
No	LFRW	82	
	PHLF	46	
Serum bilirubin (mg/dL)	LFRW	10.5 (4.5-16.9)	0.245
	PHLF	8.6 (4.7-16.7)	
Serum albumin (g/L)	LFRW	47 (32-47)	0.931
	PHLF	38.5 (34-47)	
INR	LFRW	0.95 (0.84-1.13)	0.480
	PHLF	0.96 (0.83-1.25)	
ICG R15 (%)	LFRW	7.8 (0.5-46.5)	≤0.001
	PHLF	24.6 (7.9-61.9)	
Operation time (min)	LFRW	470 (79-840)	0.478
	PHLF	455 (120-950)	
Intraoperative blood loss (mL)	LFRW	300 (40-1000)	0.246
	PHLF	400 (100-1200)	
Volume of resected liver (cm^3^)	LFRW	210 (55-1611)	0.907
	PHLF	304 (60-1360)	
Surgical method			
Left hemihepatectomy	LFRW	144 (104-248)	0.349
	PHLF	175 (124-216)	
Right hemihepatectomy	LFRW	650 (308-1148)	
	PHLF	608 (392-936)	
Extended hemihepatectomy	LFRW	1440 (1148-1568)	
	PHLF	1510 (1360-1611)	
Others	LFRW	76 (61-98)	
	PHLF	73 (60-83)	

Values are presented as *n* (%) or median (range).

*LFRW*: liver function recovered well; *PHLF*: postoperative liver dysfunction.

**Table 5:** Correlation of clinical characteristics and postoperative complications.

Factor	Group of complication	Result	*P* value
Age, years	Minor	65 (34-76)	0.728
	Moderate-to-severe	63 (48-80)	
Sex			
Male	Minor	29	0.553
	Moderate-to-severe	43	
Female	Minor	29	
	Moderate-to-severe	35	
Hepatitis			
Yes	Minor	8	0.869
	Moderate-to-severe	10	
No	Minor	50	
	Moderate-to-severe	68	
Serum bilirubin (mg/dL)	Minor	8.3 (4.5-16.9)	0.596
	Moderate-to-severe	9.0 (4.7-16.9)	
Serum albumin (g/L)	Minor	39 (32-45)	0.197
	Moderate-to-severe	40 (34-47)	
INR	Minor	0.96 (0.84-1.25)	0.667
	Moderate-to-severe	0.95 (0.83-1.13)	
ICG R15 (%)	Minor	9.6 (1.5-22.0)	≤0.001
	Moderate-to-severe	17.0 (2.7-61.9)	
Operation time (min)	Minor	433 (79-733)	0.358
	Moderate-to-severe	463 (79-950)	
Intraoperative blood loss (mL)	Minor	300 (40-1000)	0.688
	Moderate-to-severe	400 (80-1200)	
Volume of resected liver (cm^3^)	Minor	216 (61-1440)	0.462
	Moderate-to-severe	210 (60-1611)	
Surgical method			
Left hemihepatectomy	Minor	216 (104-248)	0.180
	Moderate-to-severe	144 (105-216)	
Right hemihepatectomy	Minor	395.5 (308-1148)	
	Moderate-to-severe	707.5 (338-936)	
Extended hemihepatectomy	Minor	1280 (1148-1440)	
	Moderate-to-severe	1464 (1360-1611)	
Others	Minor	77.5 (61-98)	
	Moderate-to-severe	76 (60-89)	

Values are presented as *n* (%) or median (range).

## Data Availability

The data that support the findings of this study are available on request from the corresponding author. The data are not publicly available due to privacy or ethical restrictions.

## Additional Points

*Summary*. 147 patients who scheduled for hCCA resection underwent a preoperative ICG test. Preoperative ICG R15 was significantly associated with PHLF and moderate-to-severe postoperative complications.
